The article "Bioinformatics Analysis Reveals the Related Role of miR-511-5p in the Progression of Breast Cancer" was published in 2022. Journal: J Healthc Eng.

# Bioinformatics Analysis Reveals the Related Role of miR-511-5p in the Progression of Breast Cancer

**DOI:** 10.1155/2022/7146338

**Published:** 2022-02-10

**Authors:** Teng Wang, Jinquan Liu, Rui Zhong, Yidan Zhang, Zhenxuan Sun, Jutao Li, Gang Hu, Li Sun, Jintao Liu

**Affiliations:** ^1^Department of Thyroid Surgery, Dalian Central Hospital Affiliated to Dalian Medical University, Dalian, 116033, Liaoning Province, China; ^2^Dalian Medical University, Dalian 116041, Liaoning Province, China; ^3^Department of Clinical Medicine, Datong University School of Medicine, Datong, 037008, Shanxi Province, China

## Abstract

Breast cancer remains a dangerous disease, and delving the molecular mechanism of breast cancer is still necessary. To illustrate the role of miR-511-5p, TCGA database was used to excavate the abundance of miR-511-5p, and the miR-511-5p level was measured in the pathological tissues and tumor cell lines. Moreover, the targets of miR-511-5p were identified with miRDIP and GEPIA and then were used for functional enrichment analysis. Besides, the targets of miR-511-5p were analyzed with the protein-protein interaction (PPI) network for the hub nodes, and then the expression levels of the hub nodes were visualized with the GEPIA database. The results showed that miR-511-5p was significantly downregulated in multiple types of tumor samples in the online database, and the downregulated miR-511-5p was also found in pathological tissues and tumor cell lines. Moreover, 48 genes were identified as the potential targets of miR-511-5p by miRDIP and GEPIA databases and enriched in cell cycle, PI3K/AKT, and P53 pathways. Besides, seven genes including BRCA1, FN1, CCNE1, CCND1, CHEK1, BUB3, and CDC25A were identified as the hub nodes by the PPI network, and CCNE1 and CHEK1 were confirmed to be related with the prognostic survival of the patients with breast cancer. In conclusion, the proofs in this study suggest that reduced miR-511-5p was a biomarker event for breast cancer, and CCNE1 and CHEK1 served as potential targets of miR-511-5p to involve the progression of breast cancer.

## 1. Introduction

Considerable clinical data have confirmed that breast cancer is a malignant disease which is a major cause in cancer-related death among females in the world [1, 2]. At present, radiotherapy, chemotherapy, and drug intervention have been widely used for the treatment of breast cancer, while the completely healing break cancer is still difficult [3]. Moreover, more than 60% patients have been confirmed at the middle or late stage when they first accepted the diagnosis, which seriously increases the possibility of cancer recurrence [4]. Therefore, even with the current therapeutic techniques, the outcomes of the sufferers with breast cancer remain poor. Thus, more biomarkers and the unambiguous molecular mechanism are still necessary for clinical treatment.

The article "Bioinformatics Analysis Reveals the Related Role of miR-511-5p in the Progression of Breast Cancer" was published in 2022. Journal: J Healthc Eng.

Microarray analysis of RNA abundance is an effective strategy for investigating the pathogenesis of diseases, and it has been widely used for identifying the biomarkers and drug targets of various tumors [5, 6]. MicroRNAs (miRNAs), a class of short noncoding RNAs consisting of 22 nucleotides, involve the multiple life progression of cells [7, 8]. Recently, increasing studies have indicated that the expression disorder of miRNAs is related with the formation and development of some tumors [9]. For multiple types of breast cancer, the difference in the miRNA profile of the sufferers and healthy people has been revealed by many studies, and some miRNAs have been proved as the biomarkers or key nodes in the progression of breast cancer [10, 11]. Downregulated miR-511-5p in some tumors has been observed by many studies, and miR-511-5p can effectively suppress the development of some tumors [12]. For colorectal cancer, the study has proved that miR-511-5p can block the migration and proliferation of multiple tumor cell lines. However, more proofs are necessary to illustrate the molecular mechanism in the development of breast cancer [13].

This study attempted to delve the functions and the related mechanism of miR-511-5p in the progression of breast cancer via bioinformatics analysis methods and provide some reference for breast cancer treatment.

## 2. Materials and Methods

### 2.1. The Clinical Data Analysis of The Cancer Genome Atlas (TCGA)

The clinical data about the pathological and related healthy tissues of the breast cancer sufferers were obtained from TCGA database. The abundance of miR-511-5p was obtained and visualized with TCGA data online analysis tool (https://bioinfo.life.hust.edu.cn/miR_path/index.html). Moreover, the expression levels and survival curves of the genes were obtained and visualized with the GEPIA database (https://gepia.cancer-pku.cn/).

### 2.2. Clinical Tissues

The pathological tissues and adjacent tissues of the patients were collected for exploring the expression level of miR-511-5p. This study was approved by the ethics committee of the hospital.

### 2.3. Cell Culture

The MCF-10A, MDA-MB-231, MDA-MB-468, and MCF-7 cells were purchased from Wuhan Procell Life Science & Technology Co., Ltd. (Wuhan, China). For the cell culture, all cells were cultured with Dulbecco's Modified Eagle Medium (Shanghai Hengfei Biotechnology Co., Ltd., Shanghai, China) containing 10% fetal bovine serum (Jiangsu Kewei Biotechnology Co., Ltd., Jiangsu, China) in an incubator with 37°C and 5% CO_2_.

The article "Bioinformatics Analysis Reveals the Related Role of miR-511-5p in the Progression of Breast Cancer" was published in 2022. Journal: J Healthc Eng.

### 2.4. qRT-PCR

Total RNA of the tissues or cells was treated with TRIzol reagent (Beijing Solebao Technology Co., Ltd., Beijing, China). cDNA of total RNA was prepared with the PrimeScript RT-PCR kit (Shanghai Shanran Biotechnology Co., Ltd., Shanghai, China). The reaction system was prepared following the instruction of the kit, and the abundance of miR-511-5p (forward: GTGTCTTTTGCTCTG; reverse: GTGCAGGGTCCGAGGT) was measured by qRT-PCR. Moreover, U6 (forward: CTCGCTTCGGCAGCACA; reverse: AACGCTTCACGAATTTGCGT) was selected as the endogenous controls. Finally, the abundance of miR-511-5p was calculated with the 2^−(ΔΔCt)^ method. The qRT-PCR was performed according to the following conditions: 95°C for 5 min, followed by 40 cycles of 95°C for 15 s, 62°C for 30 s, and 72°C for 30 s.

### 2.5. Gene Ontology (GO) Enrichment Analysis

The targets of miR-511-5p were predicted with miRDIP (https://ophid.utoronto.ca/mirDIP/), and then significantly upregulated genes were screened with GEPIA (https://gepia.cancer-pku.cn/). The genes in top 5% potential targets predicted by the miRDIP database were selected as the candidates. GO enrichment analysis was performed for investigating the functions of the targets of miR-511-5p. Briefly, the EntrezIDs of the targets were obtained from the DAVID database (https://david.ncifcrf.gov/). After that, the packages including topGO, clusterProfiler, and org.Hs.eg.db of R language were performed to search the related functional modules of the EntrezIDs. Moreover, the common genes of the targets and the genes in the GEPIA database were analyzed and visualized with the Venny tool (https://bioinfogp.cnb.csic.es/tools/venny/index.html).

### 2.6. Kyoto Encyclopedia of Genes and Genomes (KEGG) Enrichment Analysis

KEGG enrichment analysis was performed to observe the related pathways of the targets of miR-511-5p. In brief, the targets of miR-511-5p were enriched by the online tool of DAVID database, and then pathway modules with *p* value <0.05 were visualized with the ggplot2 package of R language.

### 2.7. Protein-Protein Interaction (PPI) Network Analysis

PPI network analysis was performed to select the hub genes in the targets of miR-511-5p, and the targets of miR-511-5p were analyzed with STRING (https://www.string-db.org/). After that, the key nodes of the datasets were analyzed and visualized with Cytoscape software.

### 2.8. Statistical Analysis

All experiments were performed at least 3 times, independently. Data analysis was performed by SPSS 20.0. Moreover, all results were handled with the chi-squared test or ANOVA with Tukey's post hoc test. *P* < 0.05 meant that the statistical significance existed in two groups.

The article "Bioinformatics Analysis Reveals the Related Role of miR-511-5p in the Progression of Breast Cancer" was published in 2022. Journal: J Healthc Eng.

## 3. Results

### 3.1. Identification of miR-511-5p in TCGA

To explore the role of miR-511-5p in breast cancer, UALCAN and TCGA data online analysis tool were used to excavate the expression of miR-511-5p in tumor samples and normal samples. The results showed that miR-511-5p was significantly downregulated in tumor samples (Figure 1).

### 3.2. miR-511-5p Was Significantly Downregulated in Breast Cancer

For verifying the role of miR-511-5p in breast cancer, the pathological samples of the patients and breast cancer cell lines were used to observe the abundance of miR-511-5p. The results showed that obviously reduced miR-511-5p was detected in breast cancer tissues and cell lines including MDA-MB-231, MDA-MB-468, and MCF-7 cells (Figures 2(a) and 2(b), *P* < 0.01). These observations supported that decreased miR-511-5p was related with the progression of breast cancer.

### 3.3. GO and KEGG Enrichment

To analyze the functions of miR-511-5p in this disease, the potential targets of miR-511-5p were obtained by the miRDIP database, and the upregulated targets were screened by the GEPIA database. The results showed that 48 upregulated genes in breast cancer samples from TCGA were selected as candidate targets of miR-511-5p (Figure 3(a)). Besides, the functions and regulation mechanism of 48 genes were identified by GO and KEGG enrichment analysis (Figure 3(a)). For GO enrichment, it was found that the eight genes including BRCA1, BRCC3, CCND1, RAD21, CHEK1, BUB3, SOX4, and CDC25A were related with the regulation of cell cycle phase transition (Figure 3(b)). For KEGG enrichment, the genes including CCND1, CCNE1, RAD21, CHEK1, BUB3, and CDC25A were related with the cell cycle, the genes including CCND1, CCNE1, COL5A2, FN1, and BRCA1 were associated with PI3K/AKT pathways, and the genes including CCND1, CCNE1, and CHEK1 were connected with P53 pathways.

### 3.4. PPI Network

To screen the key genes to reveal the regulation mechanism of miR-511-5p, selected 48 targets were analyzed with the STRING database and then visualized by Cytoscape software. The results showed that seven genes including BRCA1, FN1, CCNE1, CCND1, CHEK1, BUB3, and CDC25A were identified as the hub nodes in the targets of miR-511-5p (Figure 4).

### 3.5. The Expressions and Prognostic Functions of the Hub Nodes in Breast Cancer

To verify the expression of the hub nodes in breast cancer, the hub nodes identified by the PPI network were analyzed by the CEPIA database. The results showed that all hub nodes remarkably increased in breast cancer. However, only abundant CCNE1 and CHEK1 were significantly related with the prognostic survival rate of the patients (Figures 5 and 6). Thus, these observations suggested that CCNE1 and CHEK1 were associated with the poor outcomes of breast cancer.

The article "Bioinformatics Analysis Reveals the Related Role of miR-511-5p in the Progression of Breast Cancer" was published in 2022. Journal: J Healthc Eng.

## 4. Discussion

This study analyzed the clinical data of the patients with breast invasive carcinoma obtained from TCGA database to reveal the role of miR-511-5p, and the targets of miR-511-5p were also predicted by the miRDIP database. Moreover, the targets of miR-511-5p were identified with the GEPIA2 database, and the increased genes were then analyzed with KEGG and GO enrichment. Besides, this study investigated the protein interaction network of the selected targets, and the potential possibility of the acquired hub nodes for predicting the prognosis of the patients with breast cancer was also explored.

miRNAs play important roles in cell activities via involving the normal metabolic processes [14]. At present, accumulating research studies have proved that the disorder of miRNA could induce the malignant behaviors of multiple tumors, and targeting some key miRNAs has been increasingly thought as a promising way for cancer treatment [15, 16]. The results of this study indicated that miR-511-5p exhibited low abundance in the pathological tissues in TCGA database, and decreased miR-511-5p was also found in the breast cancer cell lines, and the result of TCGA also proved that miR-511-5p was also remarkably downregulated in some tumors. Some studies have indicated that miR-511-5p was significantly downregulated in several tumors, and it plays a tumor suppressor to inhibit the progression of cancer. Reduced miR-511-5p has also been found in lung squamous cell carcinoma, and miR-511-5p overexpression could effectively block the angiogenesis of the tumor via impeding the expression of VEGFA [17]. Thus, these proofs suggest that miR-511-5p may function as a tumor inhibitor to restrain the development of breast cancer.

miRNAs are characterized with the repressing translation of proteins via specially binding the 3'-UTR of their mRNAs. For miR-511-5p, it can impede the migration and invasion of gastric cancer via targeting PAK2 [17]. In this study, the targets of miR-511-5p were predicted by the miRDIP database, and 48 targets were significantly upregulated in tumor tissues according to TCGA database. The progression of breast cancer involves the dysfunction of multiple cellular functions and pathways [18]. In this study, it was found that the 48 targets of miR-511-5p were involved in several functional modules including the regulation of cell cycle phase transition and DNA damage checkpoint. Especially, BRCA1, BRCC3, CCND1, RAD21, CHEK1, BUB3, SOX4, and CDC25A were involved in the cell cycle, and BRCA1, BRCC3, CCND1, CHEK1, and SOX4 were involved in the DNA damage checkpoint. Due to the rapid proliferation of the cells in the progression of cancer development, the aberrant regulation of cell cycle has been confirmed as a biomarker event of cancer [19]. Inhibiting the cell cycle can effectively block the deterioration of the cancer. Repo et al. proved that suppressing the cell cycle could effectively inhibit the progression of breast cancer [20].

The article "Bioinformatics Analysis Reveals the Related Role of miR-511-5p in the Progression of Breast Cancer" was published in 2022. Journal: J Healthc Eng.

Increasing studies have indicated that the disorder of cellular signaling pathways takes part in the progression of breast cancer including malignant proliferation and invasive and metastatic behaviors. In this study, it was found that the targets of miR-511-5p were related with the cell cycle, P53 pathway, PI3K/AKT pathway, viral carcinogenesis, focal adhesion, and so on. Moreover, CCND1, CCNE1, and CHEK1 were related with P53 pathways, and CCND1, CCNE1, COL5A2, FN1, and BRCA1 were related with PI3K/AKT pathways. P53 serves as a tumor inhibitor which is inactivated or mutant in many cancer cells [21]. For breast cancer, P53 mutant has also been reported as a biomarker event, and decreased P53 has a direct connection with the poor outcomes of the sufferers [22]. PI3K/AKT pathway has been discovered in various tumors, and activated PI3K/AKT also involves in the chemoresistance and cell growth [23]. For breast cancer, inactivation of the PI3K/AKT pathway could effectively inhibit deterioration of cancer [24]. Wang et al. identified that activated PI3K/AKT induced by WWP1 upregulation can promote the chemical resistance of triple-negative breast cancer [25].

This study also investigated the key genes in the targets of miR-511-5p via PPI network analysis, and seven genes including BRCA1, FN1, CCNE1, CCND1, CHEK1, BUB3, and CDC25A were identified as the hub nodes. Moreover, this study also found that CCNE1 and CHEK1 were related with the prognostic survival rate of the patients. CCNE1 functions as a tumor supporter which was related with the poor prognosis of the patients with negative breast cancer [25]. CHEK1 also serves as an oncogene which directly affects the survival of the patients. Besides, CCNE1 and CHEK1 were proved to be related with the connection of the cell cycle and P53 and PI3K/AKT pathways. The study has also found that CCNE1 is one key gene which is enriched in P53 pathways, and the report of Zhang et al. has also suggested that circDENND2A can regulate the activity of P53 pathways in lung cancer through the miR-34a/CCNE1 axis [26, 27]. In addition, CHEK1 has been confirmed to have a direct link with P53 in colon cancer, and inhibited CHEK1 could significantly promote the apoptosis of P53-knockdown cancer cells [28].

The article "Bioinformatics Analysis Reveals the Related Role of miR-511-5p in the Progression of Breast Cancer" was published in 2022. Journal: J Healthc Eng.

## 5. Conclusion

In summary, this study suggested that miR-511-5p acts as a tumor suppressor in breast cancer, and miR-511-5p blocking the growth of breast cancer is related with the PI3K/AKT and P53 pathways.

## Figures and Tables

**Figure 1:** Expression profile of miR-511-5p from TCGA (originated from TCGA data online analysis tool).

**Figure 2:** The abundance of miR-511-5p in breast cancer tissues and cell lines. (a) The expression of miR-511-5p in normal and tumor samples. (b) The relative expression level of miR-511-5p in MCF-10A, MDA-MB-231, MDA-MB-468, and MCF-7. ^*∗∗*^*P* < 0.01.

**Figure 3:** GO and KEGG enrichment for the targets of miR-511-5p. (a) The targets of miR-511-5p in the miRDIP database and differentially expressed genes obtained from the GEPIA database. (b) GO enrichment for the identified genes. (c) KEGG enrichment for the identified genes (the larger the size, the more significant the proportion of the gene).

**Figure 4:** The PPI network of the identified genes from the targets of miR-511-5p predicted by the miRDIP database and differentially expressed genes obtained from the GEPIA database.

**Figure 5:** The expression levels of hub nodes were visualized with GEPIA. (a) BRCA1. (b) BUB3. (c) CCND1. (d) CCNE1. (e) CDC25A. (f) CHEK1. (g) FN1.

**Figure 6:** The connection of hub nodes and the survival rates of the patients were visualized with GEPIA. (a) BRCA1. (b) BUB3. (c) CCND1. (d) CCNE1. (e) CDC25A. (f) CHEK1. (g) FN1.

## Data Availability

The data used to support the findings of this study are available from the corresponding author upon reasonable request.
